RETRACTED

# Awareness and perception of malaria and dengue at school and college level in the district of Multan

**DOI:** 10.1371/journal.pone.0260868

**Published:** 2022-02-10

**Authors:** Muhammad Essa, Muhammad Ahmed Taj, Muhammad Hakim Khan, Muhammad Amjad Bashir, Hasnain Farooq, Reem A. Alajmi, Mohamed Hashem, Saad Alamri, Manal A. El-Zohri, Kaleem Ullah

**Affiliations:** 1 Medical Officer Basic Health Unit, Health Department, Talpur Kot Chuta Dera Ghazi Khan, Punjab, Pakistan; 2 Health Department, Rural Health Center 222EB, District Vehari, Punjab, Pakistan; 3 Medical Officer Rural Health Unit, Health Department, Kalur Kot, District Bakhar, Punjab, Pakistan; 4 Department of Plant Protection, Faculty of Agricultural Sciences, Ghazi University, Dera Ghazi Khan, Punjab, Pakistan; 5 Department of Environmental Sciences, University of California, Riverside, CA, United States of America; 6 Department of Forestry, Faculty of Agricultural Sciences, Ghazi University, Dera Ghazi Khan, Pakistan; 7 Zoology Department, College of Science, King Saud University, Riyadh, Saudi Arabi; 8 Botany and Microbiology Department, Faculty of Science, Assiut University, Assiut, Egypt; 9 Department of Zoology, Faculty of Sciences, Ghazi University, Dera Ghazi Khan, Punjab, Pakistan; Harran Üniversitesi: Harran Universitesi, TURKEY

## Abstract

The purpose of this study is to examine the awareness and perception of malaria and dengue fever in Multan Punjab, Pakistan while taking into account the important role of government policies and other variables. The goal of this study is to examine the awareness of students in Multan, Pakistan on malaria and dengue. This study is based on a quantitative approach of secondary evidence from scientific journals and questionnaire surveys. It is also based on observational evidence gathered in Multan Punjab Pakistan, in a field study. The survey with school children, teachers and healthcare professionals were both formal and semi-structuralize. Studies have found that malaria and dengue mainly affect children’s schooling through their absence, but can also induce brain loss and cognitive disability. In questionnaires, students were seen to have different understanding of the illness, but also to be able to serve as agents of health reform only through teachers. A sample size of 500 respondents has been selected from different colleges of district Multan Punjab, Pakistan. Correlation technique is used for the data analysis. According to our results it is concluded that the students at college level are aware of malaria and dengue diseases, but they are not capable of engaging and serving as agents for health reform. On the basis of results it is recommended that students must teach about epidemics diseases regarding how to handle these diseases.

RETRACTED

## Introduction

Malaria and dengue diseases both are considered to grow exponentially, both in regards to prevalence and mortality rates, as well as mosquito-borne illnesses that pose a global issue of public health because of ease on the globe. Malaria is the product of Plasmodium spp protozoan parasitic infection. Usually conveyed by Anopheles spp. Human diseases include Plasmodium falciparum, *Plasmodium vivax*, and *P*. *ovale* (*P*. *falciparum*) [1].

*P*.*knowlesi*, human simian parasite outbreaks are being recorded from of the mountainous regions of South-East Asia and, in unique, Borneo Island [2]. Malaria parasites in individuals are first produced and multiplied in the liver cells and even in the red blood cells (RBCs) [3].

Parasite stages are those causing clinical manifestations of malaria in an erythrocytic loop. The sexual replication of the parasite starts in the gut when the gametocytes are obtained by a female Anopheles mosquito after a blood meal. The zygote grows through the fusion of the gametocytes which leads to the sequence of the development of oocyst and sporocyst. The parasites are contained in the salivary glands as sporozoites after 10–18 days. The sporozoites are then contaminated with the next blood meal and processes are restarted [4].

In addition, Dengue fever is a mosquito-borne disease transmitted by four different serotypes of Single-Stranded RNA viruses (DEN-1, 2, 3, 4) in the Flaviviridae family. *Aedes aegypti* [5] is normally transmitted to any of those serotypes.

The normal dengue transmission cycle, analogous to malaria, resembles the cycle between humans and vectors. Even so, the dengue virus (DENV) also has a good ability to migrate from a period of livestock transfer to a human cycle. Female mosquitoes ingest the DENV which circulates in human blood while they eat. That virus instead contagionists and reproduces in the mid-intestinal mosquito. Eventually, the hemocoel and salivary glands of the mosquito get corrupted and replicated. During the following time of feeding, the virus is then transferred by the salivary gland to other humans [6].

Concurrent malaria and dengue outbreaks arise concurrently as these conditions occur in people. Although the clinical aspects of these two diseases are identical, malaria diagnosis and dengue associated diseases may be misdiagnosed or misconstrued as mono-infections [7]. Currently, a variety of malaria-dengue infections associated have been recorded from different regions of the world regarding the very first report presented in France in July 2005 [8]; While cases of malaria and dengue infections are uncommon in Asia, their clinical seriousness is seen in contrast to one of these infections alone [9].

RETRACTED

Dengue and malaria are hard to distinguish therapeutically, but their treatment is dissimilar. A delay in the establishment of adequate management, stressed elsewhere [9] could be fatal. Indeed, clinical and biological representations of incidents of co-infection vary from actual diseases and correlations of bivariate indicate more variations amongst malaria dengue and dengue rather than malaria dengue [10].

The study highlights the important challenge of malaria and dengue infections throughout the Asian region. A debate on the clinical characteristics of these competitor diseases based on studies from various countries of Asia could assist to raise awareness amongst populations, physicians, healthcare professionals, and local medical associations of the significance of these co-infections. In order to resolve this health problem, this would open the way for specific policy recommendations. Two main arthropod-borne infectious diseases in the tropical regions are malaria and dengue; just very seldom are dual infections defined [10, 11]. Data from Asian countries, especially India, have shown an obvious increase in the occurrence of simultaneous malaria and dengue infections in the past decade.

Because of the enormous percentage of individuals registered per year, vector-borne diseases (VBD) are a threat to developing countries. Overwhelming of healthcare services in poor-resource countries could result in outbreaks of VBDs like dengue and malaria [12, 13]. Dengue fever is the largest human arboreal disease spread worldwide, causing more sickness and death than all of the other aerobic diseases [14] by *A*. *aegypti* and *A*. *albopictus* mosquito. The occurrence of diseases has been growing over time in India, with hyperendemic conditions in certain states/syndicates like Delhi [15].

One of the most significant outbreaks of this disease occurred in India (99,913 cases reported and 220 deaths) in 2015, the worst of which was Delhi (15,867 cases reported; 60 dead). As dengue is, India’s with malaria is afflicted with a separate VBD. South-East Asia is heavily afflicted and 77% of the disease prevalence is in India. [16] without widely available vaccines, the risk of certain diseases may be minimized successfully with environmental protection policies paired with worker’s prevention steps [17].

Therefore, active group involvement through better awareness and health promotion activities is necessary to produce better outcomes in vector management [18, 19]. As with many health issues in society, the population’s awareness, behavior, and behaviors (KAPs) play a significant role in enforcing VBD control steps. The WHO has advocated the use of lay people as health educators in the war against common diseases.

RETRACTED

Schools include kids with a vital chance to learn regarding emerging health and endemic disorders and how to avoid them. Teachers will play a vital role in transmitting key preventive education strategies to kids and striving at a significant health predictor–health behavior. While significant, the function of school administrators as school counselors has not received much attention. Analysis of which aspects of intervention at the community level can be strengthened by supporting teachers’ health education in schools does not exist much [20].

Limited studies study has shown the role of education providers in the battle against diseases like AIDS and oral illness [21]. Consequently, aspects of intervention and community health have to be discussed that can be turned into effective prevention initiatives at the educational level by teachers.

The level of awareness, climate, and activities of the Population surrounding mosquito-borne diseases are unavoidable in establishing a sound and successful health education policy. It was agreed to conduct this analysis in the city of Rajkot with this context. Dengue fever (DF) is an infectious disease that is prevalent in the Asian subcontinent spread by *A*. *aegypti* [22]. (In recent years, the death and the morbidity connected with this has arisen as a prominent public health issue. The dengue occurrence has increased 30 times in the last 50 years, according to the World Health Organization (WHO). Globally, 50 to 100 million dengue infections have been reported to occur annually [23].

South-East Asia, comprising 52 percent of global risk, is among the DF / DHF areas with the greatest risk. Patients with DHF and dengue shock syndrome (DSS) can have as large a case-fatality rate as 44 percent. Indeed, in many urban, peri-urban, and rural regions, the issue is becoming hyper prevalent with recurrent epidemics. In several parts of India Dengue is endemic and epidemics in several parts of India are regularly recorded [24].

Vector regulation is the best way to combat dengue because there is no antidote. Unless community engagement occurs, the community’s understanding of the disease, its manner of propagation, and reproduction sites is essential to determine the effectiveness of a community-based initiative. Information, sensitivity, and study in the practice function as a population educational diagnostic. This knowledge helps initiatives set communication goals in line with increased audience involvement and demand for resources, as well as establish customized methods suited for risky socioeconomic, political, and cultural circumstances. With about 2.5 trillion people who are at risk of infecting, the global prevalence of dengue infection is increasingly growing. The WHO reports that up to 50 million illnesses are dengue every year, resulting in 500 000 hospitalizations every year. 5. About 70 percent of 5 of these cases are studied in the field of Asia Pacific.

RETRACTED

## Methodology

The study was an Ex-Post-Facto method, that covered variables that had been expressed and which could not be influenced by the investigator. The goal of this analysis was to explore the awareness and perception of malaria and dengue in school and college. The study analyzed the relationship between awareness and perception of malaria and dengue. This study explored the interaction amongst demographic (age, gender, qualifications, etc.) and awareness and perception of malaria and dengue.

This study followed a sample methodology. The questionnaire survey has been used to interpret the features, behaviors, or actions of a group from one sample to a population [25].

### Study design

As indicated [26], the study process consisted of six main stages. The first stage describes the study topic. The reason for this study initially results from several reasons, like the absence of detailed study into the perception and awareness of malaria and dengue in school and college students. The second stage defined the study problem. The theoretical and applied literatures on awareness and perception of school and college children on the topic of malaria and dengue have been thoroughly analyzed. The third stage involves study planning. In order to facilitate the necessary fieldwork, the schools, academics, and college institutions were contacted in the Multan area. The fourth stage involves collecting information and study data and the data was collected from the schools and colleges. The fifth stage involves the analysis of data that was gathered in stage four. Stage 6 includes conclusions that hopefully provide policymakers with convincing evidence in their efforts to improve the awareness and perception of malaria and dengue in schools and colleges of Pakistan.

For data collection and analysis, the study method is a selection of tools to be used. According to [26], study and learners need to choose suitable methods in order to show their ability to understand and acknowledge their subject matter. Questions surveys are carried out to identify the opinions of students, teachers, as well as staff and their controlling factors in the country in the quantitative study methodology. This approach also includes the collection of statistical data for the analysis of dengue and malaria’s awareness in schools and colleges. Statistic results are also used to evaluate awareness and perception of malaria and dengue of students.

RETRACTED

One of the methods used to collect information for this study was the questionnaire survey. In order to assess business problems regarding awareness of malaria and dengue, the survey entitled “Awareness and perception of malaria and dengue in schools and colleges” is carried out. The survey will provide relevant evidence of awareness of malaria and dengue in schools and colleges. The survey will attempt to identify the challenges and difficulties facing students in their effort to make good awareness about malaria and dengue.

A questionnaire survey will be chosen to gather all the information and data required due to the advantages and suitability of the study questions.

#### Questionnaire format

The close-ended question formats were used for the design of the questions in this survey. Besides, a formatting style Likert-scale based on five categories was also employed (Strongly disagree, disagree, neutral, agree, and strongly agree).

### Sample & sample size

The study population is composed of students in various schools and colleges in Multan. In such schools and colleges, the total population of students was around 1000+. Taking into account the essence and aims of the study, the stratified random sampling method has been used. The survey contained both boys and girls. The ethics committees of the Ghazi University Dera Ghazi Khan provide approval for the study with subject to that before completing the questionnaire, scholars got willingness from each participant (as the participants were not minors as they were the students of final years classes and senior most of their respective institutes and are able to provide willingness, no need to get permission from their parents as they all were elders) and it is recorded in form of voice and this record will be submitted in the office of ethics committee with the coordination of Director Colleges Multan Punjab, Pakistan for study purpose only.

### Instrument

The method used to gather data was the mix of questions approved for use in the review of path-goal theory. Questionnaire for this study that evaluated various units of all variables was merged to construct a detailed questionnaire (dependent, autonomous, and moderating). The final questionnaire administered comprises two sections: the first section involves demographic and personal information; the second section involves variables like awareness of malaria and dengue, perception of malaria and dengue, etc.

### Sources of data

The study centered on the students who are studying in schools and colleges of Multan.

RETRACTED

### Collection of data

Via a range of approaches, the analysis and planned utilization of the data was told to all administrators of schools and colleges. Both questionnaires provided written material about the essence of the analysis sample in addition to the descriptive guidance. Participants were instructed not to mention specific names in the report. Participants were also told that results would be measured in composite scores to protect secrecy inside the data collection so that no personal identifying details will be shared. The sharing of knowledge on methods and applications of data collection included: demonstration at various departments to clarify leadership and analysis to all managers; email and telephone calls. As the study team operated in the schools and colleges itself at the period of the data collection, professional connections have often been used for the gathering of knowledge and for making effective usage of participants. Subconsciously, the implementation of the data collection process.

### Analysis of data

In addition to the personal observations of the scholars, the obtained data was tabulated in Excel sheet and study. It was often correlational as it aimed to establish an association between distinct study variables. The interpretation of study participants was focused on all sorts of evidences. The Pearson / Product Moment correlation is ideally adapted for investigating the interaction amongst such variable [27]. The 0.05 degree of validity of all theories was checked. Data have been evaluated using the Social Science Statistical Package (SPSS-26)

## Results

The above Table 1 shows the awareness of dengue fever of students. 48.6% (243) students have dengue fever before and 47.0% shows that they don’t have dengue fever before, 4.4% are unsure about it. The table also shows that dengue fever students are more in number than other ones.

**Table 1:** Do you have dengue fever before?

	Frequency	Percent
Yes	243	48.6
No	235	47.0
Unsure	22	4.4
Total	100	100.0

The above Table 2 shows the awareness of the malaria fever of students. 50.6% of students have malaria fever before and 48.8% shows that they don’t have malaria fever before, 0.6% (3) are unsure about it. The table also shows that malaria fever students are more in number than other ones.

**Table 2:** Do you have malaria fever before?

	Frequency	Percent
Yes	253	50.6
No	244	48.8
Unsure	3	0.6
Total	100	100.0

The above table shows the students who know anyone that have malaria fever in their respective area. The students who know that have malaria fever before are 50.4% and 44.6% show that they don’t know who has malaria fever before, 5.0% (Table 3) are unsure about it. The table also shows that malaria fever students are more in number than other ones.

RETRACTED

**Table 3:** Do you know anyone who have malaria fever before?

	Frequency	Percent
Yes	252	50.4
No	223	44.6
Unsure	25	5.0
Total	100	100.0

The above table shows the students who know anyone that have dengue fever in their respective area. The students who know that have dengue fever before are 46.0% and 46.2% show that they don’t know who has dengue fever before, 7.8% (Table 4) are unsure about it. The table also shows that dengue fever students are more in number than other ones.

**Table 4:** Do you know anyone who have dengue fever before?

	Frequency	Percent
Yes	230	46.0
No	231	46.2
Unsure	39	7.8
Total	100	100.0

### Correlation analysis

The Table 5 shows the analysis outcomes; a strong correlation shows a strong agreement between the respondents. Where (important (α) > 0.05) that is to say there is no correlation between the respondents, and if ((α), < 0.05) there is substantial relation between the respondents. The correlation coefficient is shown in the table and the factors that cause malaria and dengue fever are also shown in this table. The correlation is significant at one percent level if it’s two-tailed.

**Table 5:** Shows the correlation analysis of dengue and malaria fever.

Correlations																									
		Q1	Q2	Q3	Q4	Q5	Q6	Q7	Q8	Q9	Q10	Q11	Q12	Q13	Q14	Q15	Q16	Q17	Q18	Q19	Q20	Q21	Q22	Q23	Q24
Q1	Pearson Correlation	1	.098	-.222*	.038	.087	.052	.005	-.121	.004	-.186	-.036	-.042	-.115	.022	.025	-.016	.063	-.033	-.162	-.039	-.093	.001	.209*	.003
	Sig. (2-tailed)		.330	.026	.705	.391	.606	.959	.231	.971	.064	.726	.677	.256	.826	.809	.878	.533	.748	.107	.699	.356	.995	.037	.978
Q2	Pearson Correlation	.098	1	.045	-.180	.076	.085	.060	-.026	-.149	-.097	-.126	.110	.031	-.044	.074	.047	.014	-.140	.012	-.006	-.152	-.129	-.019	.025
	Sig. (2-tailed)	.330		.657	.073	.455	.403	.551	.798	.139	.336	.213	.275	.761	.664	.462	.639	.892	.166	.909	.954	.132	.201	.850	.801
Q3	Pearson Correlation	-.222*	.045	1	.044	.017	-.031	.033	.044	-.143	-.028	.023	.087	.010	.025	-.099	.038	-.092	.015	-.018	-.188	.007	.052	.058	.058
	Sig. (2-tailed)	.026	.657		.665	.867	.757	.741	.663	.156	.781	.820	.389	.922	.806	.327	.708	.363	.883	.855	.061	.943	.606	.564	.566
Q4	Pearson Correlation	.038	-.180	.044	1	.296**	.239*	.095	.003	.085	-.005	-.180	-.011	-.227*	.021	-.015	.067	.102	.107	-.137	-.104	.193	.235*	.128	.026
	Sig. (2-tailed)	.705	.073	.665		.003	.016	.347	.974	.403	.963	.073	.912	.023	.839	.885	.511	.312	.292	.174	.305	.054	.019	.204	.799
Q5	Pearson Correlation	.087	.076	.017	.296**	1	.093	-.060	.018	.066	-.259**	.095	-.074	-.051	.207*	.035	.132	-.006	.038	-.044	-.055	.121	.146	.127	.017
	Sig. (2-tailed)	.391	.455	.867	.003		.359	.555	.863	.513	.009	.349	.463	.614	.038	.729	.191	.954	.710	.667	.589	.229	.147	.207	.869
Q6	Pearson Correlation	.052	.085	-.031	.239*	.093	1	.145	.069	-.032	-.201*	-.187	.052	-.089	-.087	.081	-.052	.000	-.164	.006	.020	-.166	-.025	.247*	.101
	Sig. (2-tailed)	.606	.403	.757	.016	.359		.151	.492	.749	.045	.063	.609	.380	.390	.424	.607	1.000	.103	.956	.846	.098	.802	.013	.319
Q7	Pearson Correlation	.005	.060	.033	.095	-.060	.145	1	.076	.066	.035	-.010	.152	-.026	-.082	-.170	.183	-.036	.096	.206*	.031	.165	-.051	-.128	.030
	Sig. (2-tailed)	.959	.551	.741	.347	.555	.151		.452	.511	.726	.922	.132	.798	.417	.090	.069	.724	.342	.040	.758	.101	.612	.203	.767
Q8	Pearson Correlation	-.121	-.026	.044	.003	.018	.069	.076	1	.090	.222*	.044	.028	.128	.020	-.122	-.011	-.051	-.006	-.066	.029	-.058	-.034	-.054	.095
	Sig. (2-tailed)	.231	.798	.663	.974	.863	.492	.452		.371	.027	.662	.782	.204	.843	.227	.913	.614	.957	.517	.773	.567	.739	.592	.345
Q9	Pearson Correlation	.004	-.149	-.143	.085	.066	-.032	.066	.090	1	-.112	.010	-.065	.064	-.025	-.052	-.088	.034	.004	.112	-.135	.062	.291**	.079	.004
	Sig. (2-tailed)	.971	.139	.156	.403	.513	.749	.511	.371		.268	.925	.519	.530	.804	.607	.386	.735	.965	.266	.181	.537	.003	.433	.965
Q10	Pearson Correlation	-.186	-.097	-.028	-.005	-.259**	-.201*	.035	.222*	-.112	1	.099	.099	.201*	-.064	-.094	-.015	-.169	.122	-.166	-.173	-.066	-.139	-.221*	-.080
	Sig. (2-tailed)	.064	.336	.781	.963	.009	.045	.726	.027	.268		.326	.325	.045	.526	.351	.885	.094	.226	.099	.085	.513	.168	.027	.430
Q11	Pearson Correlation	-.036	-.126	.023	-.180	.095	-.187	-.010	.044	.010	.099	1	-.087	.142	-.022	-.112	-.022	.094	-.009	.063	.016	.054	-.021	-.046	-.019
	Sig. (2-tailed)	.726	.213	.820	.073	.349	.063	.922	.662	.925	.326		.389	.158	.825	.266	.831	.352	.929	.534	.878	.595	.836	.647	.854
Q12	Pearson Correlation	-.042	.110	.087	-.011	-.074	.052	.152	.028	-.065	.099	-.087	1	.292**	.116	-.008	.013	-.138	-.158	.110	-.123	.025	-.137	-.040	-.122
	Sig. (2-tailed)	.677	.275	.389	.912	.463	.609	.132	.782	.519	.325	.389		.003	.251	.934	.897	.170	.117	.277	.221	.808	.175	.692	.228
Q13	Pearson Correlation	-.115	.031	.010	-.227*	-.051	-.089	-.026	.128	.064	.201*	.142	.292**	1	.053	.089	.036	-.012	-.200*	.030	-.108	-.029	-.128	-.024	-.080
	Sig. (2-tailed)	.256	.761	.922	.023	.614	.380	.798	.204	.530	.045	.158	.003		.600	.381	.719	.905	.046	.767	.287	.775	.204	.812	.429
Q14	Pearson Correlation	.022	-.044	.025	.021	.207*	-.087	-.082	.020	-.025	-.064	-.022	.116	.053	1	.141	.276**	.035	-.109	.088	.106	.074	-.085	.148	-.010
	Sig. (2-tailed)	.826	.664	.806	.839	.038	.390	.417	.843	.804	.526	.825	.251	.600		.161	.005	.731	.280	.385	.296	.462	.402	.142	.920
Q15	Pearson Correlation	.025	.074	-.099	-.015	.035	.081	-.170	-.122	-.052	-.094	-.112	-.008	.089	.141	1	-.082	.126	-.083	-.104	-.012	.043	.203*	.241*	.085
	Sig. (2-tailed)	.809	.462	.327	.885	.729	.424	.090	.227	.607	.351	.266	.934	.381	.161		.419	.210	.413	.302	.905	.668	.043	.016	.400
Q16	Pearson Correlation	-.016	.047	.038	.067	.132	-.052	.183	-.011	-.088	-.015	-.022	.013	.036	.276**	-.082	1	.179	-.177	-.085	.201*	.105	-.118	.182	.242*
	Sig. (2-tailed)	.878	.639	.708	.511	.191	.607	.069	.913	.386	.885	.831	.897	.719	.005	.419		.075	.078	.403	.045	.299	.243	.069	.015
Q17	Pearson Correlation	.063	.014	-.092	.102	-.006	.000	-.036	-.051	.034	-.169	.094	-.138	-.012	.035	.126	.179	1	.097	-.038	.232*	.142	.334**	.177	.317**
	Sig. (2-tailed)	.533	.892	.363	.312	.954	1.000	.724	.614	.735	.094	.352	.170	.905	.731	.210	.075		.338	.705	.020	.159	.001	.078	.001
Q18	Pearson Correlation	-.033	-.140	.015	.107	.038	-.164	.096	-.006	.004	.122	-.009	-.158	-.200*	-.109	-.083	-.177	.097	1	.021	.167	.192	.306**	-.183	-.165
	Sig. (2-tailed)	.748	.166	.883	.292	.710	.103	.342	.957	.965	.226	.929	.117	.046	.280	.413	.078	.338		.832	.098	.056	.002	.068	.100
Q19	Pearson Correlation	-.162	.012	-.018	-.137	-.044	.006	.206*	-.066	.112	-.166	.063	.110	.030	.088	-.104	-.085	-.038	.021	1	-.011	-.088	.029	-.235*	-.106
	Sig. (2-tailed)	.107	.909	.855	.174	.667	.956	.040	.517	.266	.099	.534	.277	.767	.385	.302	.403	.705	.832		.915	.384	.775	.019	.294
Q20	Pearson Correlation	-.039	-.006	-.188	-.104	-.055	.020	.031	.029	-.135	-.173	.016	-.123	-.108	.106	-.012	.201*	.232*	.167	-.011	1	.114	.098	.151	.103
	Sig. (2-tailed)	.699	.954	.061	.305	.589	.846	.758	.773	.181	.085	.878	.221	.287	.296	.905	.045	.020	.098	.915		.260	.332	.135	.310
Q21	Pearson Correlation	-.093	-.152	.007	.193	.121	-.166	.165	-.058	.062	-.066	.054	.025	-.029	.074	.043	.105	.142	.192	-.088	.114	1	.274**	.073	.083
	Sig. (2-tailed)	.356	.132	.943	.054	.229	.098	.101	.567	.537	.513	.595	.808	.775	.462	.668	.299	.159	.056	.384	.260		.006	.473	.410

*. Correlation is significant at the 0.05 level (2-tailed).

**. Correlation is significant at the 0.01 level (2-tailed).

RETRACTED

## Results and discussion

Malaria is a chronic public health epidemic, which has been resolved yet regulated by several initiatives. Globalized malaria has been suppressed in 113 countries; 34 middle-income countries and malaria has been eliminated in several low-income countries. In malaria-endemic areas, most low-income countries worldwide continue to track malaria. Expression Malaria tracking the effect of malaria has been considerable in low-income countries, with Sub-Saharan Africa, where 47 out of 54 countries are endemic to malaria and most of them are malaria prevention programs. Despite (IPTp), Plasmodium falciparum infection during pregnancy was a public health concern over more than 20 years ago [28], especially throughout sub-Saharan Africa. The field has 75,000 to 200,000 deaths of infants, 900,000 deliveries of LBWs as well as 10,000 deaths of mother every single year [29]. The population of Sub-Saharan Africa is between 25 as well as 30 million pregnant women at risk Sub-Saharan Africa’s high malaria incidence is well known to public health as well as global leaders, particularly amongst vulnerable populations like pregnant women and babies. Several trials have also been performed to investigate risk factors for the greater incidence of malaria morbidity and mortality in pregnant women and babies [30].

Comprehensive study was carried out on the interaction between pregnant Tanzanian women (a) SES (defined by age, education level, residence, and wealth index), (b) exposure to malaria media, (c) knowledge of signs or symptoms of Malaria, (d) perceived seriousness of malaria, as well as (e) evidence of malaria in preventive measures (knowledge of malaria signs and symptoms in the prevention of pregnancy). While testing travel, family duty as well as age, both variables had important predictors of the high dose population. The risk of high dose SP / Fansidar has been differentiated by malaria presence in the media as well as the identification of malaria signs and symptoms, and hence the knowledge of malaria prevention measures, as the wider risk of high dose groups, are the greater the increased exposure as well as knowledge of malaria in the medium or their preventive measures. The presumed severity of malaria was also able to estimate how likely it is for travel, family obligation as well as age to be among the high-dose community. The product, therefore, of perceived malaria variable seriousness obtained is in contrast to the expected the implications of this are that, in the initially expected high-dose class, pregnant women who viewed malaria almost as dire health danger were less likely. I interpret the results of this chapter, address the shortcomings of the analysis, prescribe future studies, propose social improvements as well as conclude [31].

HBM (HBM) was used as a basis to analyze the combination of women’s care study activity with independent variables: SES (in terms of age, schooling, residence, and wealth), malaria media consumption, malaria signs and symptoms known, malaria severity perceived and malaria prevention awareness. Both variables were the significant predictor of the probability of women pursuing care with SP / Fansidar doses at ANC to avoid pregnant malaria, Transportation regulation, family liability, as well as age. Six structures lead the HBM (HBM) system: (a) the vulnerable nature of real diseases, (b), the associated disease severity, (f) the advantages of health interventions, (d) the perceived obstacle to intervention, (e) the readiness to respond as well as (f) the usefulness of oneself. HBM is founded on the conviction that individuals are more likely to prevent disease if they consider that their particular interventions will prevent disease [32].

RETRACTED

HBM discusses in my study the behavior of pregnant women in their clinical behavior in the prevention of malaria during pregnancy. My results of the study are compatible with most HBM postulations. Consequently, I found that the understanding of malaria’s severity does not immediately affect the prescription of pregnant women with ANCs after checks on travel, family duty as well as age to avoid malaria. This study rather found that the high dose of 2+SP / Fansidar prescribed was less usual among those who felt malaria to be a severe health threat. Other aspects such as the availability of SES as well as malaria-related communications have contributed greatly to raising the awareness of malaria, as well as to avoiding as well as curing women who have been embarked on treatment. Pregnant women have been well trained to avoid malaria as well as their diagnosis or management techniques. As previous studies have shown, my study also found that awareness about malaria infections among women pregnant women was a major factor in their ability to pursue as well as avoid malaria [33].

The interviews as well as secondary evidence showed that malaria has multiple impacts on the schooling of children. Malaria mostly affects schooling due to absence, but it really impacts the ability of children to read. The teachers interviewed underlined the lack of malaria as a potential outcome. This can be clarified by the easier identification of absence than physiological as well as cognitive injury. If a student is missing, it is necessary to inquire to figure out why, so it’s more difficult for a student to know the real causes if it isn’t clear that the kid is suffering through paludism if he has trouble recalling things or just has learning disorders. The scale of the lessons renders monitoring all their students much tougher for such an instructor. The teachers interviewed, who visit the students often every day, claimed that malaria in Multan wasn’t really common. They saw the illness as either a concern, but only when one was afflicted (which they said was very unusual). That may be partially even though they found it difficult to monitor whether students were sick as well as absent. In one class, it was not rare for many students to demonstrate their opinions upon this disease. The teachers said that the students were acquainted with malaria, so this was false in the children’s interviews. Those wrong comments could be because they felt children understood rather than because they actually failed to acknowledge the indifference of the children [34].

RETRACTED

The study shows a varied awareness of malaria among school children as well as some apparent shortcomings, among other symptom awareness, disease effects as well as preventive measures. This is significant that the interactions of the children for malaria did not contribute to a greater understanding of the disease. The primary source of awareness for children was schools. Although primary education in Tanzania is compulsory yet most children are present, this could serve as a valuable tool to raise understanding of malaria. The study also indicates that schools as either an information source do not suffice and that other outlets, like mass media, may be significant in the distribution of knowledge through schools [35]. It is obvious that the prevalence of malaria in Multan is high just through staring at children’s awareness. Similarly, the incidence of malaria depends not only on misinformation as well as on other causes, like insecurity as well as inadequate healthcare coverage. Poverty and bad health are associated yet hard to solve, although poverty can The Ministry of Health practically relies on global assistance to provide all the population with healthcare, sufficient for the country’s healthcare facilities. It would not only be beneficial but it also affordable to include children as well as schools in the battle against malaria [36].

In order to make children health change agents, awareness is important. If teachers are happy to take part in delivering study, they will learn this expertise. The nation, the hospital as well as NGOs will need some assistance. All the participants treated malaria as just a big issue in society except for some of its students. The teachers should explain that the disorder is pervasive to help them understand the benefits of prevention in order to make kids behave as principals of health improvements. Anyone must share the responsibility for creativity in order to persuade the students. In the current crisis, an NGO is probably to provide all the required assistance for this project as there are inadequate resources available to the government. Child participation in the war against malaria is possible in Multan; however, this involves the dedication of the community. It is essential to note what has been achieved throughout the past in order to convince the benefits of creativity, to enhance children’s knowledge against Malaria as well as to involve them with agents for health improvements. It is, therefore, necessary to study whether the invention meets human needs as well as violates old customs as well as regulations, or is deemed to be non-functional (compatibility). It must be studied unless the invention is just too complicated and whether that is easy to comprehend that can be used (complexity), in order to decide whether children will serve like health improvement agents. There are two dimensions; whether the kids are able to access as well as reveal knowledge about malaria to the group. Innovation must also be tested to see if it progresses and can see the outcomes (trial ability). It may be a means of measuring creativity if we encourage a school to train its students to also become agents for health improvements and can see the impact [37].

RETRACTED

It may well be related to the normalization of the disease in the culture but rather that the disease can be seen as common in people’s daily life, that no more respondents felt malaria is really a prevalent disorder in Multan. This may be one of the reasons for the lack of awareness and also the high incidence of children. When people don’t really see malaria as just a threat, prevention steps are not likely to be interpreted as well as the infection cannot be minimized as well as prevented without intervention [38].

With a 99 percent standard deviation, the average findings of the analysis were important. This study promotes its use of illustration as a means to increase awareness, to enhance mindset as well as to increase the ability to reduce contact among mosquitoes as well as to minimize mosquito-breeding sites throughout the form of dengue campaigns. These pieces of evidence are therefore inadequate to infer the effect on the frequency of dengue fever [39].

Identifying these procedures for dengue campaigns could be a successful means of achieving this audience Recruitment has provided a study sample divided equally amongst men and women. There were more fifth-graders, usually accompanied by fourth-grader, but instead three. It might reflect the reticence of the third-grader, assuming that, while the processes have been clarified, they may continue to read/read ratings. In reality, it can also be circulated as a whole and, furthermore, the data has not been compiled, and remains uncertain. The students either at camp are not compiled. The study of free time hobbies has found that more people preferred homework, more than shockingly, computer games as well as television. Such high-profile occasions would include participating in films, churches, diving, and athletics. The dengue cartoon, for instance–, can be played in the film theatre, screening can be given through homework, or just a church initiative can be carried out. After all, Costa Rica, its video game named Pueblo Pitanga: Enemigos Silenciosos (Pitanga VI: Silent Enemy), has been adopted by the World Health Organization as well as Pan American Health Organization, emphasizing safe water quality methods to avoid dengue [40].

RETRACTED

The majority of the respondents asked whether they knew of dengue fever. Just five had learned of dengue fever among the 54 participants. For the five, the knowledge source was as continues to follow: one student, one school; one student, TV/radio; 1 respondent, health worker; 1 respondent had not reported where they had learned about DF, as well as 1 respondent had written on the Web. However, only two interviewees indicated that mosquitoes were known to be a concern. These details suggest a determined vector epidemic, but nearly no dengue fever awareness. The HBM notes that the respondents are susceptible to mosquitoes. In combination with this instructional illustration, they may feel "perceived gravity," "perceived advantages" as well as "perceived challenges" while they understand what measures to take. They can also feel That the whole environment is a great time for constructive preparation. The expectation for contact has also shown that the population tends to provide information through the internet. That method of contact has been almost omitted from either the options list, although in the age group it was perceived to be an unusual option. Social networking should be used as an important method of targeting this population in future promotions. Such studies cannot be extended, through fact, to the creation of societies. In determining the accuracy of the study of the information portion, multiple considerations should be weighed. Second, a one-time sample was planned for the [41] sample, instead of a pretest/posttest. Throughout the "side effects" as well as "breeding" section, each survey questions demonstrated an incorrect response when uncontrolled, and even in the "transmission" segment, an uncontrolled reply was right. That was most likely responsible for an exceptionally large pre-test / post-test disparity in symptoms as well as a comparatively minor propagation disparity. Its classification of ignition has also generated substantial improvements in pre-to-posttest performance, following these structure shortcomings. In future experiments, this may be dealt with by adjusting the issue in order to correct as well as incorrect equivalent numbers of unregulated responses. The simple inclusion of the "I don’t know" option may otherwise be necessary to improve the precision of the ratings. Throughout the Keeping as well as Activities areas, legitimacy was improved while the responses were not accurate or incorrect; in the Mindset portion, as well as stuff is done, respondents clearly showed whether they thought in the Activities portion [42].

RETRACTED

Secondly, a study published for adults in [40] was conducted with adolescents. While certain improvements have been made to content/language, the issue retains nuanced as well as mature. However, children have been able to achieve high ratings and enhance the general reliability of the graphics. The effectiveness of the mechanism in general and/or its consistency of the graphics, in particular, can be related to this [43].

The findings revealed that respondents’ conduct about DF was substantially changed, via an understanding of the fact that perhaps the disorder was severe as well as action should be done to help avoid it. The mindset of respondents against their efforts to support deter DF has undergone an incredibly dramatic shift. The HBM notes that risk assessment is key to behavioral change. In addition, compartmental changes are driven by "cues to behavior," that must be carried out in an environment. in addition to improvement. The evident All such criteria are discussed in tandem with explicitly specified as well as defined protections. In addition, leadership theory suggests children would like to collaborate among adults as well as multiple study affirm that children are capable reform actors [44].

While most people (> 50 percent) have sufficient knowledge of such DF in the sample, their reproductive areas of the dengue vector were not completely identified. People infected with dengue from ’dirty sites, like drains and trash, in which larvae from other mosquitoes were observed. Each views of people about breeding sites are markedly hierarchical. There are actually three symptoms of dengue: DF, DHF as well as dengue shock syndrome. But in both of them, fever is perhaps the most frequent cause. The lack of awareness of DF obtained from this study compares to the above observed in related study on KAP in India and, except for a few that have observed fever to be apparent signs, most participants have not been able to precisely classify DF’s classic signs. Jamaica, Pakistan as well as Thailand were also the signs most commonly documented in related studies in India [45].

The study participants were presumably unable to claim the standard DF signs hadn’t encountered the illness directly or observed a situation from a nearby associate or just a member of the group. The low understanding of DF signs in the study population can easily be interpreted with some other typical explanations for fever, including measles, typhoid, and so on. Although the information gap was not statistically significant between the rural and urban regions. There was insufficient knowledge of vector reproduction as well as biting intentions. Most interviewees stated the mosquitoes transferring DF races in drains as well as waste (67%) although less than half the participant’s stagnant water. Mostly in the morning (58 percent) as well as evening (44 percent), over half of the participants record mosquito bite [46]. This is associated with some recent study, which found that most people were conscious whether dengue vectors could be morseling after sunrise or sunset typically throughout all homes, in huge container containers like the metal / plastic buckets, concrete tanks, and cisterns, people stored water for bathing/ potable water. Many small containers are most often used to gather water as well as to store water while there was insufficient water supply, for example, in metal / plastic containers. These containers were suitable breeding grounds for Anopheles’ mosquito when kept without even a proper jar lid for just an extended time. Throughout this report, almost all (81 percent) of HHS conduct water storage in tanks, and around 40% store water in small proportions made of plastic as well as steel. The waste created either by the municipal squad was seen daily or alternately in most places, and yet people were indiscriminately throwing the waste out of their homes [47].

RETRACTED

In short, most people in Pondicherry have inadequate knowledge of dengue fever, how it is spread, how the habitat of vector breeding, as well as the action of mosquito biting. The prevention activities in household containers and frequent parts were poor against Anopheles mosquito breeding. Another big explanation for the rising trends in dengue in this densely populated urban area may be the lack of basic population awareness of dengue epidemiology as well as vector bionomics [48].

## Conclusion

In Multan, children are aware of malaria today, but they are not capable of engaging and serving as agents for health reform. If teachers are able to give awareness to pupils, with the support of the government, the hospital, or an NGO, children have the ability to help deter the spread of malaria into their communities. This is possible because the workers of hospitals saw the children as key players in fighting malaria and that almost all respondents thought that malaria was a significant social concern.

RETRACTED

## Supporting information

S1 File Questionaire of the study. (PDF)

S2 File All data in addition information. (XLSX)
